This article has been retracted.

# miR-26a-5p mediates TLR signaling pathway by targeting CTGF in LPS-induced alveolar macrophage

**DOI:** 10.1042/BSR20192598

**Published:** 2020-06-04

**Authors:** Chunyan Li, Tingfeng Han, Run Li, Liming Fu, Lei Yue

**Affiliations:** 1 Department of Emergency, Luoyang Central Hospital Affiliated to Zhengzhou University, Luoyang 471000, He’nan Province, China; 2 Department of Gynecology, Luoyang Central Hospital Affiliated to Zhengzhou University, Luoyang 471000, He’nan Province, China

**Keywords:** connective tissue growth factor, miR-26a-5p, severe pneumonia, toll-like receptor signaling pathway

## Abstract

To explore the regulation mechanism of miR-26a-5p and connective tissue growth factor (CTGF) in lipopolysaccharide (LPS)-induced alveolar macrophages, which is a severe pneumonia cell model. MH-S cells were grouped into Normal group, Model group, negative control (NC) group, miR-26a-5p mimic group, oe-CTGF group, miR-26a-5p mimic + oe-CTGF group. The expression level of miR-26a-5p, CTGF and Toll-like receptor (TLR) signaling related molecules (TLR2, TLR4 and nuclear factor-κB p65) were detected by qRT-PCR and WB, respectively. The cell viability and apoptosis rate were detected by methyl thiazolyl tetrazolium (MTT) and flow cytometry, respectively. Compared with the Normal group, the expression level of miR-26a-5p was significantly decreased, while CTGF protein level was significantly increased in the Model group. Compared with the Model group, MH-S cells with miR-26a-5p overexpression showed enhanced cell viability, decreased apoptosis rate, declined expression level of TLR signaling related molecules and reduced level of tumor necrosis factor-α (TNF-α), interleukin (IL) 6 (IL-6) and IL-1β, while those with CTGF overexpression had an opposite phenotype. In conclusion, miR-26a-5p can inhibit the expression of CTGF and mediate TLR signaling pathway to inhibit the cell apoptosis and reduce the expression of proinflammatory cytokines in alveolar macrophages which is a cell model of severe pneumonia.

## Introduction

Severe pneumonia, also known as toxic pneumonia or fulminant pneumonia, is a severe disease in clinical respiratory medicine, with rapid progress, high incidence and critical conditions [1]. Severe pneumonia was mostly caused by bacterial infection [2]. The patients show dyspnea, cough and expectoration, gastrointestinal bleeding and other symptoms, while severe cases even appear with sudden shock, diffuse intravascular coagulation, organ failure etc. In recent years, the prevalence of severe pneumonia increased by years, bringing serious economic burden to the patients and their families.

Currently, the main clinical treatment for severe pneumonia is antibiotics, but it is only effective to the patients in the early stage, therefore, timely administration of antibiotics can save the lives of patients to a large extent. However, the increase in pathogenic bacteria resistance gradually worsens the efficacy of antibiotics, so it is necessary to further explore more effective treatments of severe pneumonia [3]. In addition to early diagnosis and treatment, the key to severe pneumonia treatment is to improve the patients’ immune function, namely, to regulate the immune function of patients to achieve effective anti-inflammation [4]. Alveolar macrophages are mainly distributed in the respiratory tract and alveolar surface, which are the most important regulatory cells in local inflammatory microenvironment and inflammatory response in the lung, serving as the first line of defense against invasion of foreign substances [5]. Therefore, we used alveolar macrophages to explore the new treatment of severe pneumonia in vitro.

Connective tissue growth factor (CTGF) is a member of the highly conserved ccN polypeptide family and is involved in cell proliferation, development, adhesion, migration, angiogenesis etc. Moreover, CTGF can predict prognosis and its expression is associated with the development of a variety of cancers [6]. Studies have also confirmed that CTGF is involved in fibrotic lesions in lung tissue, which is highly expressed in transplanted lung tissue, while normal lung has no expression [7]. MicroRNAs (miRNAs) are a class of single-stranded RNAs with a length of approximately 21 bases [8]. Numerous studies have found that miRNAs play an important role in the maintenance of cell function by acting on targeted genes, so as to get involved in the regulation of organ development, cell apoptosis, proliferation and differentiation [9]. Among them, miR-26a-5p is significantly correlated with the development of lung cancer [10,11]. Moreover, CTGF is the possible target gene of miR-26a-5p.

Toll-like receptors (TLRs) play an important role in tissue damage repair, tissue damage-induced inflammation and tumor progression, while alveolar macrophages, as an important regulatory cell of inflammation, is closely related to severe pneumonia [12,13].

In the present study, a severe pneumonia model was established by lipopolysaccharide (LPS)-stimulated mouse alveolar macrophages *in vitro*. And we found that miR-26a-5p negatively regulated CTGF to mediate TLR pathway, so as to participate in the development of severe pneumonia, hoping to provide more new ideas for the treatment of severe pneumonia.

## Materials and methods

### Cell culture

The MH-S cells (mouse alveolar macrophages) used in this experiment were purchased from the ATCC cell bank of the United States and cultured with RPMI 1640 medium (Gibco, U.S.A.) containing 10% fetal bovine serum and 100 μg/ml streptomycin (Beijing Reagan Biotechnology Co., Ltd.) and 100 U/ml penicillin (Beijing Reagan Biotechnology Co., Ltd.) in an incubator with 5% CO_2_ at 37°C. Cells in logarithmic growth phase were taken for further experiments.

### Cell grouping, transfection and model establishment

The cells were divided into six groups, Normal group (normal cells without any treatment), Model group (only stimulated with 1 μg/ml LPS for 12 h), negative control (NC) group (transfection with negative plasmids and stimulated with 1 μg/ml LPS for 12 h), miR-26a-5p mimic group (transfected with miR-26a-5p overexpression plasmids and stimulated with 1 μg/ml LPS for 12 h), oe-CTGF group (transfected with CTGF overexpression plasmids and stimulated with 1 μg/ml LPS for 12 h), miR-26a-5p mimic + oe-CTGF group (co-transfected with miR-26a-5p and CTGF overexpression plasmids and stimulated with 1 μg/ml LPS for 12 h). The interest plasmids were purchased from Vigenebio. Transfection was performed by using the Lipofectamine 2000 (Invitrogen) kit. Briefly, 4 μg of the target plasmid and 10 μl of Lipofectamine 2000 were diluted with 250 μl of Opti-MEM medium (Gibco), respectively, and the solutions were gently mixed. After standing at room temperature for 5 min, the two solutions were mixed together and stand for 20 min, and then the mixture were added to the cell culture wells. The plate was gently shaken to mix the culture medium, and then placed in a cell culture incubator for 6 h. Then the medium was replaced by fresh complete medium. Cells were harvested for subsequent experiments at 36 or 48 h after transfection.

### Double luciferase reporter assay

The binding site of miR-26a-5p and CTGF was predicted using target gene prediction software. The CTGF 3′UTR sequence containing the target (CTGF-WT) was artificially synthesized, and the WT target site was subjected to site-directed mutagenesis using the QuikChange II® Site-Directed Mutagenesis kit (Stratagene, La Jolla, CA, U.S.A.) to obtain a mutant sequence (CTGF-MT). CTGF-WT and CTGF-MT recombinant plasmids were obtained by inserting the synthetic target gene fragments WT and MT into the pmiR-RB-REPORTTM (Guangzhou Rui Bo Biotech Co., Ltd.), respectively, which were co-transfected into HEK 293T cells with miR-26a-5p mimic plasmid or mimic control plasmid, respectively. After transfection for 48 h, the cells were collected, lysed, centrifuged for 3–5 min to obtain the supernatant. The luciferase assay kit (RG005, Beyotime Biotechnology Co., Ltd., Shanghai, China) was used to measure luciferase activity according to the instructions. Luciferase assay buffer and firefly luciferase assay solution were prepared. Then 100 μl of buffer solution was mixed with substrate (1:100) to prepare luciferase assay working solution. Subsequently, 100 μl of working solution were added into 20–100 μl of sample and the firefly luciferase activity was measured. Cells transfected with empty vectors was set as a blank control. Relative luciferase activity = firefly luciferase/*Renilla* luciferase. The experiment was repeated three times.

### qRT-PCR

Total RNA was extracted by TRIzol (15596026, Invitrogen, Carlsbad, CA, U.S.A.) method. The integrity of RNA was identified by 1% agarose gel electrophoresis, and the concentration and purity of RNA were measured by spectrophotometry. Reverse transcription experiments were carried out in accordance with the instructions of the PrimeScript RT reagent kit (RR047A, Takara, Japan). Primers for miR-26a-5p, TLR2, TLR4, nuclear factor-κB (NF-κB) p65, U6 and GADPH were designed and synthesized by Shanghai Biotech (see Table 1). Real-time quantitative PCR was performed on 7500 ABI (U.S.A.) according to the instructions of SYBR®Premix Ex Taq™ II kit (of TaKaRa, Dalian, China) with a reaction system of 20 μl:10 μl SYBR Premix, cDNA template 2 μl, upstream and downstream primers each 0.6 μl and DEPC water 6.8 μl. The reaction conditions were set as initial denaturation at 95°C for 30 s, denaturation at 95°C for 30 s, annealing at 55°C for 20 s, extension at 72°C for 30 s, 40 cycles. The amount of expression of each gene in the cell is calculated by 2^−ΔΔ*C*_t_^, which indicates the ratio of the expression of the target gene in the experimental group and the control group using the following formula: Δ*C*_t_ = *C*_T__(target gene)_ − *C*_T__(internal reference)_, ΔΔ*C*_T_ = Δ*C*_t__experiment group_ − Δ*C*_t__control group_. miR-26a-5p uses U6 as an internal reference, and other genes use GAPDH as an internal reference.

**Table 1:** qRT-PCR primer sequence

Gene name	Forward primer (5′–3′)	Reverse primer (5′–3′)
*miR-26a-5p*	CGCGAATTCTTGAGGTGAGGCTCAGGAGG	ACGGGATCCTTGGCTACAGGCAAAGGGTT
*TLR2*	GTCTTTCACCTCTATTCCCTC	GTCTCTACATTTCCTATCCTG
*TLR4*	TTCAGAGCCGTTGGTGTATC	CCCATTCCAGGTAGGTGTTT
*NF-κB p65*	GCATCCAACCTGAAAATCGTG	CCCCAAATCCTTCCCAAACT
*U6*	TGCGGGTGCTCGCTTCGGCAGC	CCAGTGCAGGGTCCGAGGT
*GADPH*	TGGTGAAGGTCGGAGTGAAC	GGAAGATGGTGATGGCCTTTC

### Western blot

Cells were collected and lysed by RIPA solution (P0013B, Beyotime Biotechnology Biotechnology Co., Ltd, Shanghai, China) containing phenylmethylsulfonyl fluoride and protein phosphatase inhibitor (Thermo Fisher Scientific, U.S.A.). After being shaken and suspended, the cells were incubated on ice for 30 min, followed by centrifugation at 12000 rpm at 4°C for 10 min. The protein concentration was determined by BCA protein quantitative kit (Thermo Fisher Scientific, U.S.A.) and adjusted to 4 g/l by PBS. Then 30 g of extracted total protein was separated by SDS/PAGE and transferred to nitrocellulose membrane and sealed with 5% skim milk-TBST for 1.5 h. Subsequently, CTGF rabbit monoclonal antibody (1:1000, ab209780, Abcam, U.K.), TLR2 rabbit polyclonal antibody (1:1000, ab209217, Abcam, U.K.), TLR4 rabbit polyclonal antibody (1:1000, ab13556, U.K.), NF-κB p65 rabbit polyclonal antibody (1:500, ab16502, Abcam, U.K.), GAPDH rabbit monoclonal antibody (1:10000, ab181602, Abcam, U.K.), were added on to the corresponding NC membranes, respectively, which were incubated at 4°C overnight. Next day, the membranes were rinsed with TBST for 15 min for three times and incubated with diluted sheep anti-rabbit secondary antibody (1:20000 to 1:50000, ab205718, Abcam) at room temperature for 90 min. After that, the membranes were rinsed with TBST again and developed by ECL luminescence reagent and photographed by SmartView Pro 2000 (uvci-2100, Major Science, U.S.A.). Quantity One software was used for protein band grayscale scanning, and statistical analysis was performed after comparing the gray value of experimental groups with that of GAPDH.

### Methyl thiazolyl tetrazolium test

The cell viability of each group was detected by methyl thiazolyl tetrazolium (MTT) cell proliferation and cytotoxicity test kit (C0009, Beyotime Biotechnology, Shanghai, China). Briefly, the transfected cells were seeded in a 96-well plate, and each experimental group was treated with 1 μg/ml of LPS for 12 h, then 10 μl of MTT solution (5 mg/ml) was added to each well and the plates were incubated for 4 h in the incubator. Subsequently, 100 μl of Formazan lysate (Gibco, U.S.A.) was added to each well, and the mixture was incubated at 37°C until the formazan was completely dissolved under light microscope, and the absorbance was measured at 570 nm. Cell viability = (absorbance of experimental group − absorbance of blank control group)/(absorbance of normal control group − absorbance of blank control group).

### Flow cytometry

The apoptosis rate was detected by Annexin V-FITC Apoptosis Detection Kit (C1063, Beyotime Biotechnology, Shanghai, China). After transfection for 24 h, cells were washed with pre-cooled PBS and centrifuged at 2000 rpm/min for 5 min at room temperature twice. Then 300 μl of Binding Buffer were added to resuspend the cells. Subsequently, 5 μl of Annexin V-FITC and 10 μl of propidium iodide (PI) were added and the mixture was incubated on the ice for 15 min with dark surroundings. Flow cytometry was performed on Cube6 (Partec, Germany) and the excitation wavelength was 480 nm. FITC was detected at 530 nm and PI was detected at the wavelength greater than 575 nm.

The cell cycle was detected by cycle detection kit (C1052, Beyotime Biotechnology, Shanghai, China). Collected cells (1 × 10^6^) were centrifuged at 1500 rpm/min for 10 min. Each sample was resuspended by 2 ml of PBS and centrifuged again. After discarding the supernatant, the cells were fixed with 1 ml of pre-cooled 75% ethanol at 4°C overnight. Next day, the cells were washed with pre-cooled PBS twice to remove the fixative. PI staining solution was prepared, which contained 500 μl of staining buffer, 25 μl of PI staining solution (20×), 10 μl of RNaseA (50×). The cells were gently resuspended with 500 μl of PI staining solution, incubated at 37°C for 30 min in the dark and detected by flow cytometry at 4°C in the dark.

### ELISA

The cells were seeded in 24-well plates, transfected and treated with LPS. The supernatant was collected, in which the inflammatory factors, interleukin (IL) 6 (IL-6), tumor necrosis factor-α (TNF-α) and IL-1β were determined according to the instructions of ELISA test kit (R&D, U.S.A.). A standard curve was drawn, and the level of inflammatory factors in each group was calculated.

### Statistical analysis

Data analysis and processing were performed by SPSS 21.0 software (SPSS, Inc, Chicago, IL, U.S.A.). All measurement data were expressed as mean ± standard deviation. Comparison among groups was performed using one-way ANOVA and post-hoc Bonferroni test. *P*<0.05 showed that the difference was statistically significant.

## Results

### miR-26a-5p targets and regulates the expression of CTGF

The TargetScan website showed a targeted binding relationship between miR-26a-5p and CTGF (Figure 1A). The luciferase activity in the miR-26a-5p mimic and CTGF-WT co-transfected group was significantly lower than that in the NC group (*P*<0.05). The intensity of luciferase activity in the miR-26a-5p mimic and CTGF-MUT co-transfection group had no significant difference compared with the control group (*P*>0.05, Figure 1B). These results indicate that miR-26a-5p can target and regulate CTGF gene expression.

**Figure 1:** Bioinformatics prediction and double luciferase reporter assay for the targeting relationship between miR-26a-5p and CTGF (**A**) The bioinformatics website predicts the binding site between miR-26a-5p and CTGF. (**B**) Double luciferase reporter assay validates the targeting relationship between miR-26a-5p and CTGF. Compared with the miR-NC group, *P<0.05.

### Expression of miR-26a-5p in each group

The expression of miR-26a-5p in each group of cells was detected by qRT-PCR (Figure 2). The results showed that compared with the Normal group, the expression levels of miR-26a-5p in the other groups were significantly down-regulated (all *P*<0.05). Compared with the Model group, the expression level of miR-26a-5p were significantly up-regulated in the miR-26a-5p mimic group and the miR-26a-5pmimic + oe-CTGF group (both *P*<0.05). There was no significant difference in the expression of miR-26a-5p between Model, NC group and oe-CTGF group (*P*>0.05).

**Figure 2:** miR-26a-5p expression level in each group Compared with the Normal group, *P<0.05. Compared with the Model group, ^#^*P*<0.05. Compared with the NC group, ^$^*P*<0.05. Compared with the miR-26a-5p mimic group, ^&^*P*<0.05. Compared with the oe-CTGF group, ^@^*P*<0.05.

### miR-26a-5p reversely regulates the expression of CTGF induced by LPS

The CTGF protein expression level in each group of cells were detected by WB (Figure 3). Compared with the Normal group, the expression of CTGF protein in the other groups was significantly up-regulated (all *P*<0.05). Compared with the Model group, the expression of CTGF protein was significantly down-regulated in the miR-26a-5p mimic group, which was significantly up-regulated in the oe-CTGF group (all *P*<0.05). Compared with the oe-CTGF group, the expression of CTGF in the miR-26a-5p mimic + oe-CTGF group was significantly down-regulated (*P*<0.05). There was no significant difference in CTGF protein expression level among the Model group, the NC group and the miR-26a-5p mimic + oe-CTGF group (*P*>0.05). These results indicate that miR-26a-5p can inhibit the expression of CTGF in MH-S cells stimulated by LPS.

**Figure 3:** WB detection of CTGF protein expression in each group of cells (**A**) Protein band diagram. (**B**) Statistical graph of protein expression. Compared with the Normal group, *P<0.05. Compared with the Model group, ^#^*P*<0.05. Compared with the NC group, ^$^*P*<0.05. Compared with the miR-26a-5p mimic group, ^&^*P*<0.05. Compared with the oe-CTGF group, ^@^*P*<0.05.

### miR-26a-5p protects the cell viability inhibited by LPS

The cell viability of each group of cells was detected by MTT assay (Figure 4). Compared with the Normal group, the cell viability of the other groups was significantly decreased (all *P*<0.05). Compared with the Model group, the cell viability was significantly increased in the miR-26a-5p mimic group, which was significantly decreased in the oe-CTGF group (all *P*<0.05). Compared with the oe-CTGF group, the cell viability of the miR-26a-5p mimic + oe-CTGF group was significantly increased (*P*<0.05). There was no significant difference in cell viability among the Model group, the NC group and the miR-26a-5p mimic + oe-CTGF group (*P*>0.05).

**Figure 4:** MTT detection of cell viability in each group of cells Compared with the Normal group, *P<0.05. Compared with the Model group, ^#^*P*<0.05. Compared with the NC group, ^$^*P*<0.05. Compared with the miR-26a-5p mimic group, ^&^*P*<0.05. Compared with the oe-CTGF group, ^@^*P*<0.05.

### miR-26a-5p reduces cell apoptosis and cells G_0_/G_1_ phase caused by LPS

Apoptosis rate in each group of cells was detected by flow cytometry (Figure 5A,B). Compared with the Normal group, the apoptosis rate in the other groups was significantly increased (all *P*<0.05). Compared with the Model group, the apoptotic rate was significantly decreased in the miR-26a-5p mimic group, which was significantly increased in the oe-CTGF group (all *P*<0.05). Compared with the oe-CTGF group, the apoptosis rate of miR-26a-5p mimic + oe-CTGF group was significantly decreased (*P*<0.05). There was no significant difference in the percentage of apoptosis among the Model group, the NC group and the miR-26a-5p mimic + oe-CTGF group (*P*>0.05).

**Figure 5:** Flow cytometry to detect cell apoptosis and cell cycle in each group of cells (**A**) Flow cytometry detected cell apoptosis in each group. (**B**) Statistical results of apoptosis rate in each group. (**C**) Flow cytometry detected cell cycle in each group. (**D**) Statistical results of cell cycle distribution in each group. Compared with the Normal group, *P<0.05. Compared with the Model group, ^#^*P*<0.05. Compared with the NC group, ^$^*P*<0.05. Compared with the miR-26a-5p mimic group, ^&^*P*<0.05. Compared with the oe-CTGF group, ^@^*P*<0.05.

Cell cycle results were shown in Figure 5C,D. Compared with the Normal group, the proportion of cells arrested in the G_0_/G_1_ phase was increased in the other groups (both *P*<0.05), and the proportion of cells distributed in the S and G_2_/M phases decreased. Compared with the Model group, the proportion of cells in the G_0_/G_1_ phase was decreased in the miR-26a-5p mimic group, which in the oe-CTGF group was significantly increased (both *P*<0.05). Compared with the oe-CTGF group, the proportion of cells in the G_0_/G_1_ phase of the miR-26a-5p mimic + oe-CTGF group was significantly lower (*P*<0.05). There was no significant difference in the cell cycle distribution among the Model group, the NC group and the miR-26a-5p mimic + oe-CTGF group (*P*>0.05).

### miR-26a-5p inhibits the expression level of TLR signaling pathway up-regulated by LPS

To verify whether miR-26a-5p and CTGF regulate TLR signal pathway in the mouse alveolar macrophage severe pneumonia model, qRT-PCR and Western blot were used to detect the expression level of TLR2, TLR4 and NF-κB in each group of cells (Figures 6 and 7). ELISA was used to detect the expression levels of pro-inflammatory factors, TNF-α, IL-1β and IL-6, which are the downstream molecules of TLR signaling pathway (Figure 8).

**Figure 6:** qRT-PCR detection of TLR2, TLR4, NF-κB expression level (**A**) mRNA expression level of TLR2. (**B**) mRNA expression level of TLR4. (**C**) mRNA expression level of NF-κB. Compared with the Normal group, *P<0.05. Compared with the Model group, ^#^*P*<0.05. Compared with the NC group, ^$^*P*<0.05. Compared with the miR-26a-5p mimic group, ^&^*P*<0.05. Compared with the oe-CTGF group, ^@^*P*<0.05.

**Figure 7:** Western blot detection of TLR2, TLR4, NF-κB expression (**A**) Protein band diagram. (**B**) Statistical graph of protein expression levels. Compared with the Normal group, *P<0.05. Compared with the Model group, ^#^*P*<0.05. Compared with the NC group, ^$^*P*<0.05. Compared with the miR-26a-5p mimic group, ^&^*P*<0.05. Compared with the oe-CTGF group, ^@^*P*<0.05.

**Figure 8:** ELISA detects the expression levels of TNF-α, IL-1β and IL-6 in each group (**A**) Expression level of TNF-α. (**B**) Expression level of IL-1β. (**C**) Expression level of IL-6. Compared with the Normal group, *P<0.05. Compared with the Model group, ^#^*P*<0.05. Compared with the NC group, ^$^*P*<0.05. Compared with the miR-26a-5p mimic group, ^&^*P*<0.05. Compared with the oe-CTGF group, ^@^*P*<0.05.

Compared with the Normal group, the expression levels of TLR2, TLR4 and NF-κB genes and pro-inflammatory factors (TNF-α, IL-1β and IL-6) in the other groups were significantly increased (all *P*<0.05). Compared with the Model group, the expression levels of TLR2, TLR4 and NF-κB as well as pro-inflammatory factors were significantly decreased in the miR-26a-5p mimic group, which were were significantly increased in the oe-CTGF group (all *P*<0.05). Compared with oe-CTGF group, the expression levels of TLR2, TLR4 and NF-κB as well as pro-inflammatory factors in miR-26a-5p mimic + oe-CTGF group was significantly lower (*P*<0.05). There was no significant difference in TLR2, TLR4 and NF-κB as well as pro-inflammatory factors expression levels among the Model group, NC group and miR-26a-5p mimic + oe-CTGF group (*P*>0.05).

## Discussion

Numerous researches have confirmed that miRNAs play important roles in pneumonia or lung injury-related diseases [14–16]. By regulating the secretion of inflammatory factors such as IL-6 in the mononuclear macrophage system, miR-492 can play a role in the infection and pathogenesis of *Mycoplasma pneumoniae* [17]. In addition, some researchers found that miR-155 can significantly attenuate the inflammatory response of acute lung injury in mice when investigating the effect of miRNA on acute lung injury induced by LPS [18]. Our study is the first one reporting the targeting and negatively regulating relationship between miR-26a-5p and CTGF.

In our study, cell viability was increased, and cell apoptosis rate was inhibited in MH-S cells with miR-26a-5p overexpression, while in those with CTGF overexpression, the results showed opposite trends. CTGF is widely expressed in many human tissues and organs, which is essential for normal lung development and gets involved in the cell proliferation and differentiation, the regulation of extracellular matrix production, the vascular development etc. [19]. Study from Bogatkevich et al. demonstrated the importance of CTGF in lung tissue repair and fibrosis [20]. Fehrholz et al. found that the high expression level of CTGF induced by glucocorticoids had adverse effects on long-term remodeling of lung cells, which can be reversed by the combination use of caffeine which can promote the recovery of lung homeostasis [21]. In addition, CTGF has the effect of inducing apoptosis [22–24]. Our results consisted of the findings of above literatures, suggesting that miR-26a-5p negatively regulated CTGF to inhibit apoptosis of alveolar macrophages.

Meanwhile, we also found that miR-26a-5p mediates the TLR signaling pathway, so as to inhibit the apoptosis of mouse alveolar macrophages. Moreover, miR-26a-5p overexpression is associated with the reducing the expression level of pro-inflammatory factors TNF-α, IL-6 and IL-1β. Previous studies have also confirmed that the TLR signaling pathway is closely related to immune recognition and inflammatory response. The abnormality of TLR signaling pathway may cause related diseases and lead to adverse effects [25]. NF-κB is a critical downstream molecule in TLR signaling pathway. When TLR is stimulated by pathogenic microorganisms, it activates NF-κB to induce the release of inflammatory factors to initiate the innate immunity [26]. TLRs mediate the activation of related signaling enzymes mainly through two pathways: dependent on myeloid differentiation factor 88 (MYD88) pathway and non-dependent MYD88 pathway [27]. The activation of the TLR signal causes transcriptional expression of inflammatory mediators and increased expression of NF-κB and MAPK, which in turn activates the natural immune system and the acquired immune system, so as to regulate gene expression of various mediators of immune and inflammatory to clear pathogens and infected cells [28–30]. Therefore, miR-26a-5p can inhibit TLR signaling by inhibiting CTGF expression, so as to reduce the expression of related pro-inflammatory factors in mouse alveolar macrophage.

In conclusion, miR-26a-5p can specifically inhibit CTGF expression, mediate TLR signaling pathway to inhibit apoptosis and reduce pro-inflammatory factor TNF-α, IL-6, IL-1β expression of LPS-induced mouse alveolar macrophages MH-S cells. However, the present study did not observe how CTGF activates the TLR signaling pathway, and the specific mechanism of CTGF-induced apoptosis needs further exploration in the future.

## Abbreviations

CTGF: connective tissue growth factor
IL: interleukin
LPS: lipopolysaccharide
miRNA: microRNA
MTT: methyl thiazolyl tetrazolium
MYD88: myeloid differentiation factor 88
NC: negative control
NF-κB: nuclear factor-κ B
PI: propidium iodide
TLR: toll-like receptor
TNF-alpha: tumor necrosis factor-α
